The article "Valproic acid attenuates intercellular adhesion molecule-1 and E-selectin through a chemokine ligand 5 dependent mechanism and subarachnoid hemorrhage induced vasospasm in a rat model" was retracted in 2023. Reasons: duplicated images; overlap with earlier publications; unreliable data; concerns about the data.

# Valproic acid attenuates intercellular adhesion molecule-1 and E-selectin through a chemokine ligand 5 dependent mechanism and subarachnoid hemorrhage induced vasospasm in a rat model

**DOI:** 10.1186/s12950-015-0074-3

**Published:** 2015-04-02

**Authors:** Chih-Zen Chang, Shu-Chuan Wu, Chih-Lung Lin, Aij-Lie Kwan

**Affiliations:** Department of Surgery, Faculty of Medicine, School of Medicine, Kaohsiung Medical University, Kaohsiung, Taiwan; Division of Neurosurgery, Department of Surgery, Kaohsiung Medical University Hospital, No.100, Tzyou 1st Road, Kaohsiung, Taiwan; Department of Surgery, Kaohsiung Municipal Ta Tung Hospital, Kaohsiung, Taiwan

**Keywords:** Chemokine ligand 5, Intercellular adhesion molecule–1, Subarachnoid hemorrhage, Vasospasm, Vascular cell adhesion molecule–1, Valproic acid

## Abstract

**Background:**

Up-regulation of regulated upon activation, normal T-cell expressed and secreted (RANTES/CCL5) and adhesion molecules is observed in the serum of animals following experimental subarachnoid hemorrhage (SAH). The present study was to examine the effect of valproic acid (VPA) on RANTES and alternation of adhesion molecules in this model.

**Methods:**

A rodent SAH model was employed. Animals were randomly assigned into six groups. Basilar artery (BA) was harvested for intercellular adhesion molecule-1 (ICAM-1), vascular cell adhesion molecule–1 (VCAM-1), and E-selectin evaluation (western blotting) and RANTES (rt-PCR). 1 ng CCL5 recombinant protein intrathecal injection was performed in the VPA + SAH groups. (N = 5).

**Results:**

Convoluted internal elastic lamina, distorted endothelial wall, and smooth muscle micro-necrosis was prominently observed in the SAH groups, which is absent in the VPA treatment and the healthy controls. Treatment with VPA dose-dependently reduced the ICAM-1, E-selectin and RANTES level, compared with the SAH group (p <0.01). The administration of CCL5 significantly increased CD45(+) glia and ICAM-1 level in the VPA treatment groups.

**Conclusion:**

VPA exerts its anti-vasospastic effect through the dual effect of inhibiting RANTES expression and reduced adhesion molecules. Besides, VPA also decreased CD45(+) cells transmigrated to the vascular wall. The administration of CCL5 significantly reversed the inhibitory effect of this compound on CD45(+) monocytes, E-selectin, and ICAM-1 level. This study also lends credence to support this compound could attenuate SAH induced adhesion molecules and neuro-inflammation in a CCL5 dependent mechanism.

**Electronic supplementary material:**

The online version of this article (doi:10.1186/s12950-015-0074-3) contains supplementary material, which is available to authorized users.

The article "Valproic acid attenuates intercellular adhesion molecule-1 and E-selectin through a chemokine ligand 5 dependent mechanism and subarachnoid hemorrhage induced vasospasm in a rat model" was retracted in 2023. Reasons: duplicated images; overlap with earlier publications; unreliable data; concerns about the data.

## Background

Delayed neurological deficit, and acute cerebral ischemia associated with subarachnoid hemorrhage (SAH) induced vasospasm persists to be a major cause of mortality and disability in patients suffered from ruptured aneurysm [1-4]. Owing to the lack of adequate medical treatment for this condition, it prompts many pre-clinical and clinical studies of the disease content [5-7]. There is a mounting body of both direct and circumstantial evidence that spasmogenic substances or ligands are critical in the development and maintenance of cerebral vasospasm. Basic molecular and cellular research also implicates two major hypotheses as key points to cerebral vasospasm. One hypothesis centers on the synergic roles of nitric oxide, a potent vasodilator, nitric oxide synthase and endothelin-1, a strong endogenous vaso-constrictor, all released form endothelial cells once SAH happened [8-13], and the other focuses on intracellular signal transduction [4,5,9,14-21]. The putative importance of inflammatory activity has not been fully emphasized, even its role in the genesis of cerebral vasospasm has been recognized. Till now, various inflammatory constituents, including adhesion molecules, cytokines, leukocytes, immunoglobulins, and complements, were observed in the pathogenesis of SAH induced brain injury and delayed cerebral vasospasm [9,11,18,22-28].

The blood clot and its by-product, existed in the subarachnoid space, are able to induce innate and delayed sterile inflammation, which mediates subsequent acute arteries and arteriolar constriction, passive venous obliteration and delayed arterial spasm [21]. However, the benefits of inflammation development after SAH remains unclear. CC chemokine ligand-5 (CCL5), or regulated on activation, normal T-cell expressed, and secreted (RANTES), is expressed by cell types such as T-cells, fibroblasts, and mesangial cells [22]. Through interacting with specific chemokine receptors (CCR1, CCR3, CCR4, and CCR5) [17,29-32], RANTES is able to mediate monocytes and T-cells transmigration into the vascular intima [17,33]. Glass et al. demonstrated monoclonal antibody for CCL5 was able to diminish leukocyte infiltration into the central nervous system and reduced neurologic deficit in a multiple sclerosis mice [30,31]. It may be reasonable to postulate that RANTES is involved in inflammation in the brain and plays a putative role in SAH induced vaso-constriction.

It is well known that leukocyte migration into the endothelium of postcapillary venous was mediated by a cascade of events initiated by the selectin family of adhesion molecules [5,14,23,34]. The adhesion glycoproteins family, including intercellular adhesion molecule-1 (ICAM-1), vascular CAM-1 (VCAM-1) and E-selectins, plays a major role in the formation of firm adhesion and transendothelial migration of leucocytes into inflamed vessels. Both ICAM-1 and VCAM-1 are expressed on cerebral vascular endothelial cell lines derived from the human, and can be up-regulated by pro-inflammatory cytokines, such as tumor necrosis factor alpha (TNF-α) or interleukin-1(IL-1), involving activation of nuclear factor κ-light-chain-enhancer of activated B cells (NF-κB) and activator protein 1 (AP-1) [14,35,36].

The article "Valproic acid attenuates intercellular adhesion molecule-1 and E-selectin through a chemokine ligand 5 dependent mechanism and subarachnoid hemorrhage induced vasospasm in a rat model" was retracted in 2023. Reasons: duplicated images; overlap with earlier publications; unreliable data; concerns about the data.

Valproic acid (VPA, 2-propylpentanoic acid), a histone deacetylase (HDAC) inhibitor, is widely used in the treatment of epilepsy [37-39]. In addition to its anti-epilepsy effects, VPA has been shown to mediate neuroprotection through the activation of signal transduction pathways, such as the extracellular signal-regulated kinase (ERK) pathway and through inhibiting proapoptotic factors [40]. Like other HDAC inhibitors, VPA has been shown to inhibit histone deacetylases and leads to the accumulation of acetylated histones and acetylated proteins, which is crucial for the regulation of gene expression by chromatin remodeling [11,37,41,42]. Recent studies were focused on its chronic inflammatory effect in sporadic amyotrophic lateral sclerosis, Alzeimer’s disease, Huntington’s disease and Parkinson’s disease [43,44].

Taking these findings together, we propose that VPA, with its unique property in gene expression, may be effective in SAH-induced inflammation and vasospasm. Given the importance of arterial lesion formation and the various effects of pro-inflammatory cytokines stimulation on leukocyte and endothelial dysfunction, the rat SAH model was used to test the hypothesis that VPA can attenuate RANTES associated late onset inflammation following experimental SAH. The suppression of adhesion molecules can partly attribute to its inhibitory effect on the following systemic immunity subsequent to SAH.

## Methods

### Materials

Valproic acid (VPA) is characterized as a potent inhibitor of histone deacetylases and was bought from the Sigma-Aldrich China Inc. Shanghai 20031, China. Polyclonal anti-rat intercellular adhesion molecule-1 (ICAM-1, MBS246106), vascular CAM-1 (VCAM-1, MBS190465) and E-selectins (MBS343017) antibody were obtained from MyBioSource, Inc. San Diego, CA 92195–3308, USA. Recombinant CC chemokine ligand-5 (CCL5), or regulated on activation, normal T-cell expressed, and secreted (RANTES, MBS143280) protein was purchased from MyBioSource, Inc. San Diego, CA 92195–3308, USA. CNM protein extraction kits were from Biochain (K3012010, Hayward, CA 94545, USA). An osmotic mini-pump was bought form Alzet corp, Palo Alto, CA 94306, USA. VPA was prepared by Ms. Wu SC (Kaohsiung Medical University Hospital, Kaohsiung 807, Taiwan), and phosphate-buffered saline (PBS, bought from Sigma-Aldrich China Inc. Shanghai 20031, China) was used as a vehicle.

The article "Valproic acid attenuates intercellular adhesion molecule-1 and E-selectin through a chemokine ligand 5 dependent mechanism and subarachnoid hemorrhage induced vasospasm in a rat model" was retracted in 2023. Reasons: duplicated images; overlap with earlier publications; unreliable data; concerns about the data.

### Induction of experimental SAH

Fifty four male Sprague–Dawley rats (n = 9), weighing between 300–400 g (purchased from the BioLasco Taiwan Co., Ltd., authorized by Charles River Lab), were used in this study. All experimental protocols were approved and supervised by the University of Kaohsiung Medicine Animal Research Committee and in accordance with the Declaration of Helsinki (1964). The rats received anesthesia by an intraperitoneal injection of a mixture of 0.9 mg/100 gm xylazine and 5.5 mg/100 gm KetaVed. 1 ml/kg body weight (BW) fresh arterial blood was withdrawn from tail artery and injected into the craniocervical junction using a stereotactic apparatus (Stoelting, Wood Dale, IL 60191, USA) [45]. No mortality was found during the study. After the induction, animals were placed in ventral recumbent position for 30 minutes to let ventral blood clot formation. The repeated induction was performed 48 hr after the 1^st^ induction. After monitoring for respiratory distress and giving mechanical ventilation if necessary, the animals were returned to the vivarium till fully awake. A habitat was offered with a 12 h light–dark cycle and an access to food and water ad lib.

### General design of experiments and treatment groups

The animals were randomly divided into the following groups (9 rats/group): 1) sham operated (no SAH); 2) SAH only; 3) SAH plus vehicle; SAH rats receiving VPA treatment of 4) 10 mg/kg/day, 5) 20 mg/kg/day and 6) 40 mg/kg/day. Treatment group was defined as animals received VPA administration 1 h after the induction of SAH. The dosage was adjusted according to our pilot study, devoid of hepatic and renal toxicity. The first administration of VPA was intraperitoneal injection at 1 h after induction of SAH and then by using an osmotic mini-pump (Alzet corp, Palo Alto, CA 94306, USA). PBS was used a vehicle. After re-anesthesia, CSF sampling from each animal was obtained through a 30-gauge needle into the foramen magnus by using stereotactic apparatus (Stoelting, Wood Dale, IL 60191, USA). The animals were sacrificed by perfusion–fixation 72 h after 2nd SAH. Cortical tissue homogenates were obtained by means of placing a 22-gauge needle inserted, 3 mm in depth, into the skull bone (N = 5) through a burr hole craniectomy (2 mm apart from the bregma). To test the neuro-inflammatory effect of VPA, another experiment was carried out in the the 40 mg/kg/day VPA + SAH group with 7) 1 ng CCL5 recombinant protein intrathecal injection or 8) not (5 animals each group). The tissues were frozen instantly and cut into 25 μm-thick sections (Reichert-Jung Ultracut E ultramicrotome). They were then stained with hematoxylin and eosin for video-assisted microscopy and the analysis of BA cross-sectional area.

The article "Valproic acid attenuates intercellular adhesion molecule-1 and E-selectin through a chemokine ligand 5 dependent mechanism and subarachnoid hemorrhage induced vasospasm in a rat model" was retracted in 2023. Reasons: duplicated images; overlap with earlier publications; unreliable data; concerns about the data.

### Perfusion–fixation

At the end of experiment, the rats were anesthetized by administration of 7 mg/kg Zoletil 50 (a mixture of tiletamine hypochloride and zolazepam hypochloride. VIRBAC, L.I.D., 06516 Carros, France). The femoral artery was catheterized to obtain blood samples for arterial blood gas, Na^+^, K^+^, glutamate oxaloacetate transaminase (GOT), glutamate pyruvate transaminase (GPT), blood urea nitrogen (BUN), Creatinine (Cr) levels evaluation. Via opening the thorax, the left ventricle was canalled with a NO16 catheter with the descending aorta clamped, and the right atrium opened. 100 mL of 70 mm Hg of 0.01 M phosphate buffer (pH 7.4) was under perfusion, followed by fixation with 160 mL 2% paraformaldehyde in the PBS solution at 36°C under a perfusion pressure of 100 mm Hg. The harvested brain was immersed in a fixative at 4°C overnight. Formed subarachnoid clots covered the basilar artery (BA) was inspected in all SAH animals visually.

### Hemodynamic measurements

By using a tail-cuff method (SC1000 Single Channel System, Hatteras Instruments, NC, 27518, USA) and rectal thermometer (BIO-BRET-2-ISO. FL 33780, USA), heart rate, blood pressure, and rectal temperature of the rats were monitored before and after VPA treatment as well as at interval of 12 h after SAH.

### Neurological assessment

A modified limb-placing tests (MLPT) [42], comprised two parts: ambulation and placing/stepping reflex examinations were performed to examine the forelimb and hind-limb activity before and after animals subject to SAH, were used to evaluate the behavior change of rats before and at 24 h after the induction of SAH. The final index was the sum of the scores of walking with lower extremities and placing/stepping reflex. A motor deficit index (MDI) was calculated for each rat at each time interval. MDI score more than three were considered to be paraplegic, whereas MDI score less than three were considered neurological deficit.

### Tissue morphometric studies of basilar artery (BA)

Five selected cross-sections from the BA of each animal were randomly analyzed by two investigators blinded to the treatment groups. Automated measurements of the luminal cross-sectional area were made using computer-assisted morphometry (Image 1, Universal Imaging Corp. Downingtown, PA 19335, USA). Areas of five cross-sections from a given animal were averaged to provide a single value for each animal. Group data are expressed as the means ± standard deviation of the means.

The article "Valproic acid attenuates intercellular adhesion molecule-1 and E-selectin through a chemokine ligand 5 dependent mechanism and subarachnoid hemorrhage induced vasospasm in a rat model" was retracted in 2023. Reasons: duplicated images; overlap with earlier publications; unreliable data; concerns about the data.

### Immunostaining of microglia and astrocytes with CD45 antibodies

Video-assisted microscope (x 400, DSX500, Yuan Li Instrument Co., Ltd. 114 Taipei, Taiwan. authorized by Olympus Scientific Solutions Americas Inc. MA 02453, USA) was used to identify CD45 positive microglia and astrocytes. Isolated rat BAs were under perfusion and fixation with 4% paraformaldehyde. Coronal sections of the BAs were stored overnight on slides at −80°С in accordance with the supplier’s instructions. Mouse anti-rat CD45 monoclonal antibody (Thermo Fisher Scientific Inc. Waltham, MA 02451, USA) was used at a dilution of 1:1000, and immunostaining was performed for 40 min at 25°С and let dry overnight as described in the mouse monoclonal alkaline phosphatase anti-alkaline phosphatase (APAAP) technique [43,46]. Five consecutive sections of each rat were photographed, and the CD45 positive cells were measured.

### Immuno-histological assays for ICAM-1, VCAM-1, E-selectin, and RANTES

The BA homogenates concentrations of ICAM-1, VCAM-1, E-selectin, RANTES by using commercially available enzyme-linked immunosorbent assay kits (SOMA Acoustic Co., Ltd. Chung Hsiao E. Road, 10655 Taipei, Taiwan distributed by R&D Systems) as stated by the supplier’s instructions. Samples containing 30 μg of protein was stirred with LDS sample buffer (contains 40% glycerol, 4% lithium dodecyl sulfate (LDS), 0.8 M triethanolamine-Cl pH 7.6, 4% Ficoll®-400, 0.025% phenol red, 0.025% coomassie G250, 2 mM EDTA disodium, NuPAGE® LDS Sample Buffer (4×) NP0007; Invitrogen, Carlsbad, CA 92008, USA) and then obtained after loaded for 8% sodiumdodecyl sulfate-polyacrylamide gel electrophoresis (SDS-PAGE) and then separated after centrifuged at 12,000 rpm for 10 min. The sampling was mounted onto a polyvinylidene difluoride membrane and incubated in blocking buffer (5% non-fat dry milk in Tris-buffered saline with 0.2% Tween 20) at room temperature. Rabbit anti-rat sICAM, sVCAM, sE-selectin and RANTES polyclonal antibodies (1:1000, MyBioSource, Inc. San Diego, CA 92195–3308, USA) were coated on the walls of micro-titer plate wells. A secondary antibody conjugated with horseradish peroxidase (HRP) in TBS-t at room temperature for 1 hr. Optical densities were measured by an enhanced Pierce chemiluminescent image analyzer (a GS-700 digital densitometer, GMI, Ramsey, MN 55303, USA).

### Statistical analysis

Data are expressed as the means ± standard deviation. For group comparisons, all statistical analyses were determined with the Mann–Whitney U test (Table 1), one-way analysis of variance (ANOVA), and the Bonferroni post hoc test (Figures 1, 2, 3, 4, 5 and 6). Difference, at a probability value less than 0.01, was considered significant.

The article "Valproic acid attenuates intercellular adhesion molecule-1 and E-selectin through a chemokine ligand 5 dependent mechanism and subarachnoid hemorrhage induced vasospasm in a rat model" was retracted in 2023. Reasons: duplicated images; overlap with earlier publications; unreliable data; concerns about the data.

**Table 1:** **Modified limb-placing test (MLPT)**

**Group Treatment**	**Ambulation**	**Placing/stepping reflex**	**MDI**
**Sham-operated**	0	0	0
**SAH**	1.44 ± 0.42	1.42 ± 0.12	2.86 ± 0.36
**SAH+ Vehicle**	1.40 ± 0.20	1.42 ± 0.21	2.82 ± 0.41
**SAH+ Valproic acid**			
**10 mg/kg**	1.14 ± 0.24	0.84 ± 0.15	1.98 ± 0.39
**20 mg/kg**	1.16 ± 0.33	0.72 ± 0.25*	1.88 ± 0.58
**40 mg/kg**	0.50 ± 0.25*	0.52 ± 0.24*	1.02 ± 0.48*

Results are expressed as the mean ± SEM, n = 9; *: p < 0.01 versus SAH condition by Mann-Whitney U test.

**Figure 1:** **Comparison of lumen cross-sectional areas of the basilar artery.** Top panel: representative micrographs of the cross-section of basilar artery obtained from the sham operated rat **(A)**, SAH only animals **(B)**, the vehicle-treated SAH rats **(C)**, SAH rat treated with 10 mg/kg/day valproic acid (VPA) **(D)**, 20 mg/kg/day VPA treatment SAH rats **(E)** and 40 mg/kg/day VPA treatment in SAH animals **(F)**. Standard bar = 200 μm. Bottom panel: quantification of the lumen cross-sectional areas. All values are mean ± SD (n = 9). Valproic acid, in 40 mg/kg/day, exerted a potential to alleviate the vasospastic response when compared with the vehicle + SAH group. *, **, ***: P < 0.01 compared with the SAH group.

**Figure 2:** **Bar graph depicting VPA on the change of CD45 positive monocytes or microglia infiltrating in the wall of basilar artery after the induction of SAH.** Toppanel revealed the sham-operated animals **(A)**, the SAH group **(B)**, 10 mg/kg/day VPA treatment in SAH rats **(C)** and Treatment with 40 mg/kg/day VPA in the SAH animals **(D)**. Lower panel revealed the CD45(+) cell count among the experimental groups. Data in the figure are presented as mean ± SD (n = 9). *: P < 0.01, and #, ##: P > 0.01 when compared with the SAH group.

**Figure 3:** **Bar graph demonstrating valproic acid (VPA) on the expression of ICAM-1, VCAM-1 and E-selectin protein (western blot).** Top panel represents SAH only animals **(A)**, the vehicle-treated SAH rats **(B)**, SAH rat treated with 10 mg/kg/day valproic acid **(C)**, 20 mg/kg/day VPA treatment SAH rats **(D)** and 40 mg/kg/day VPA treatment in SAH animals **(E)**. VPA is able to decrease the expression of ICAM-1 (at a high dose), and E-selectin (at a high dose), but does not decrease SAH induced VCAM-1 expression. The ICAM-1, VCAM-1 and E-selectin expression in the SAH group was set at 100%. All values are mean ± SD. *: P < 0.01, and #, ##, ###: P > 0.01, compared with the SAH group.

The article "Valproic acid attenuates intercellular adhesion molecule-1 and E-selectin through a chemokine ligand 5 dependent mechanism and subarachnoid hemorrhage induced vasospasm in a rat model" was retracted in 2023. Reasons: duplicated images; overlap with earlier publications; unreliable data; concerns about the data.

**Figure 4:** **Level of expressed RANTES in the SAH rats receiving VPA treatment (western blotting).** Lower panel: left column bar graph revealed the adhesion molecules level in the 48 h after the induction of SAH; right column revealed the RANTES activation was late-onset inflammatory reaction, which was significantly reduced in the 40 mg/kg/day VPA treatment by the end of double shot SAH study. All groups are identical to those shown in the legend of Figure 3. Data are showed as mean ± SD. (*: P < 0.01, and #, ##,###: P > 0.01).

**Figure 5:** **The effect of CCL5 on CD45(+) cells (western blot).** Upper panel: immune-staining with CD45 monoclonal antibody. SAH animals received 40 mg/kg/day VPA treatment **(A)** and both 1 ng CCL5 intra-thecal treatment and 40 mg/kg/day VPA treatment **(B)**. CCL5 administration increased the CD45(+) cell transmembranous migration into the wall of basilar artery. N = 5. Data in the figure are presented as mean ± SD. (*,**: P < 0.01, #:P > 0.01, indicates comparison between SAH rats treatment with 40 mg/kg/day VPA or not, respectively).

**Figure 6:** **Level of expressed adhesion molecules in the SAH rats receiving VPA and CCL5 treatment (western blotting).** Upper panel: SAH rats **(A)**, SAH animals received 40 mg/kg/day VPA treatment **(B)** and both 1 ng CCL5 intra-thecal treatment and 40 mg/kg/day VPA treatment **(C)**. Bar graph revealed CCL5 reversed the effect of 40 mg/kg/day VPA on adhesion molecules. Data are showed as mean ± SD. (*: P < 0.01, and #, ##: P > 0.01).

## Results

### General observation

By the end of the study, there were no significant differences in the physiological parameters recorded, including GOT, GPT, BUN, Cr, pH, blood pressure and arterial blood gas analysis among all experimental groups. It proved that VPA in the selected dosage has a number of pleiotropic effects, devoid of hepatic and renal toxicity. Grossly, the animals in the SAH only and SAH plus vehicle groups revealed withdrawal behaviors, direction disorientation, and decreased appetite.

### Neurological deficit

A summary score of MLPT in the SAH groups were significantly higher than the healthy controls and VPA groups. The values of MDI in the SAH and SAH + vehicle groups were 2.86 ± 0.36 and 2.82 ± 0.41, respectively, compared with a score of 0 and 1.02 ± 0.48 in the healthy control and 40 mg/kg VPA, respectively. Treatment with VPA significantly improved the MDI in the SAH groups (Table 1). Likewise, paraplegia rate (defined as MDI ≥ 3 in each group) was substantially decreased in the VPA treatment groups when compared with the SAH animals.

### Cross-sectional areas of BAs

The cross-sectional areas of BAs in SAH rats were significantly reduced (Figure 1). The mean cross-sectional areas of BAs in the SAH only and SAH plus vehicle groups were reduced by 56 and 53%, respectively, when compared with the control group. VPA dose-dependently reduced the mean cross-sectional area in those animals was similar to that in controls (p > 0.01; Figure 1). The protective effect of 40 mg/kg VPA achieved statistical significance when a comparison was made with the SAH only or SAH plus vehicle group (p < 0.01).

The article "Valproic acid attenuates intercellular adhesion molecule-1 and E-selectin through a chemokine ligand 5 dependent mechanism and subarachnoid hemorrhage induced vasospasm in a rat model" was retracted in 2023. Reasons: duplicated images; overlap with earlier publications; unreliable data; concerns about the data.

### Immunostaining of microglia and monocytes with CD45 antibodies

CD45(+) astrocytes and monocytes infiltrating into the adventia are esteemed as a sign of chronic inflammation. Significant immunostaining of CD45 (LCA) cells was observed in the vascular wall of the SAH and vehicle-treatment SAH group (Figure 2). The CD45(+) cell number was counted 1.2 ± 0.5, 8.3 ± 1.4, 7.8 ± 2.3, 7.4 ± 2.6, 6.8 ± 3.1 and 4.3 ± 2.4 in the sham-operated, SAH, SAH+ vehicle, 10 mg/kg VPA + SAH, 20 mg/kg VPA treatment SAH and 40 mg/kg VPA + SAH groups, respectively. (p < 0.01, Figure 2, bottom panel). CD45(+) cells infiltration into vascular wall were increased in the CCL5 administration in 40 mg/kg/day VPA treatment SAH group (P < 0.01, Figure 5, left column).

### The expression of ICAM-1, VCAM-1, and E-selectin protein

To evaluate the leukocyte transmembrane migration into brain blood barrier and its facilitating protein in animals subjected to SAH, western blotting was used to examine ICAM-1, VCAM-1 and E-selectin. Upregulation of VCAM-1 levels in animals after the induction of SAH, no significant difference was observed among the SAH, SHA and vehicle and 10 mg/kg, 20 mg/kg and 40 mg/kg VPA plus SAH groups (Figure 3). Treatment with 40 mg/kg VPA significantly decreased the levels of E-selectin after SAH (p < 0.01) when compared with that of SAH plus vehicle group. Levels of ICAM-1 in the SAH only and SAH plus vehicle groups were elevated when compared with that of the control group and high dose VPA treatment SAH group (Figure 3, p < 0.01). In this study, VPA significantly reduced the level of E-selectin (at a high dose) and ICAM-1 (at a high dose), when compared with that of SAH group (Figure 3, p <0.01). Intrathecal administration CCL5 significant induced the suppression effect of VPA on ICAM-1 levels (Figure 6, P > 0.01).

### RANTES expression

RANTES was demonstrated to play a pivotal role in the onset of neuro-inflammation. The expression of RANTES protein was significantly induced in the SAH groups (SAH only, treatment with vehicle, 10 mg/kg and 20 mg/kg VPA) when compared with the normal controls (Figure 4. p < 0.01). VPA (at high dose) significantly decreased RANTES expression when compared with the SAH groups (P <0.01).

The article "Valproic acid attenuates intercellular adhesion molecule-1 and E-selectin through a chemokine ligand 5 dependent mechanism and subarachnoid hemorrhage induced vasospasm in a rat model" was retracted in 2023. Reasons: duplicated images; overlap with earlier publications; unreliable data; concerns about the data.

## Discussion

In this SAH study, VPA, a HDAC inhibitor, has shown to be able to attenuate SAH induced chronic inflammation. VPA were demonstrated as a novel class of potentially therapeutic agents in the treatment of epileptic seizures and bipolar disorder [38,42,43]. In the study of spinal cord injury, VPA was proved to be able to promote the proliferation and differentiation of endogenous and exogenous neural stem cell, which leads to the restoration of hind limb function and axonal remodeling [32,39]. In Shein et al’s study, VPA treatment significant reduced cerebral infarct volume, suppressed microglial activation and inhibited inflammatory markers in a permanent middle cerebral artery infarct [40]. In vitro, VPA was demonstrated to attenuate the secretion of TNF-α and IFN-γ from reactive helper T cells and monocytes in the appearance of lipopolysaccharide (LPS) [42,44]. Although the relationship between HDAC inhibitor and its protective effects remains unclear, VPA has a potent effect on the neuro-inflammation cannot be over-emphasized. A large number of in vitro and in vivo studies have revealed that HDAC inhibitor has a potent ability to stimulate neurite growth in primary cultured hippocampal neurons as well as promote axonal regeneration in animal models. By up-regulating glial cell-derived neurotrophic factor (GDNF) and brain-derived neurotrophic factor (BDNF) gene transcription in astrocyte and glioma cells located in prefrontal cortex, VPA exerts neuroprotective effect in case of CNS insults [40]. In this study, VPA was proved to be able to suppress ICAM-1(dose-dependently) and E-selecin (at high dose), which initiated the transmemebrane migration of leukocytes; by the way, activated RANTES protein level was reduced in the 40 mg/kg/day VPA treatment SAH group.

Leukocyte common antigen (LCA), also known as CD45, belongs to a family of five glycoproteins (MW 180–240 kD) which present on the surface of most T-lymphocytes [46]. The mouse anti-rat CD45 immunoglobulin was employed to detect T-lymphocytes as well as Kupffer cells. Microglia can also be perceived with anti-LCA antibodies. In this study, the expression of LCA surface marker gathered at the muscular layer of BA in the SAH rats [47]. Treatment with 40 mg/kg/day VPA significantly reduced CD45(+) lymphocytes and microglia in the SAH induced chronic vasospasm, which indicates VPA, at a selected dosage, is able to alleviate T-cell related chronic inflammation at the cellular basis.

Our previous study revealed increased adhesion molecules and pro-inflammatory cytokine in cerebrospinal fluid (CSF) after experimental aneurysmal SAH [14]. However, the relationships among the development of inflammatory response, vascular constriction, and delayed cerebral ischemia in the brain after SAH need to be clarified. In the initial of SAH, the up-regulation of ET-1 peaks 3–4 days after SAH followed by a negative feedback through activation of endothelial nitric oxide synthetase (eNOs) depletes NO, which mediated a Na^+^-K^+^ channel and further resulted in vasodilation [11,17]. Bowman et al. reported a polyclonal IL-6 antibody was able to alleviate vasoconstriction in a femoral artery SAH study [1]. The cumulative evidences support that the surge of pro-inflammatory cytokines is antecedent to radiographic vasospasm (peak at 4th to 14th days after SAH), and attenuation of cytokines tends to minimize vascular constriction and reduced cerebral ischemia [4]. The selectins, belong to transmembrane glycoproteins, are expressed on activated vascular endothelium (E-selectin), activated platelets (P-selectin), and leukocytes (L-selectin), and modulate the early adhesion interactions between endothelium and circulating neutrophils [34]. Some studies elicit elevation of levels of E-selectin, ICAM-1, and VCAM-1 in the CSF of patients after aneurysmal SAH, and E-selectin levels were severely elevated in patients with moderate or severe vasospasm [10,21,27,36]. In this study, we have found E-selectin levels to be increased in animals subjected to SAH compared with control animals. High dose VPA significantly reduced the production of E-selectin after SAH in this study.

The article "Valproic acid attenuates intercellular adhesion molecule-1 and E-selectin through a chemokine ligand 5 dependent mechanism and subarachnoid hemorrhage induced vasospasm in a rat model" was retracted in 2023. Reasons: duplicated images; overlap with earlier publications; unreliable data; concerns about the data.

Among the adhesion molecules, members of the immunoglobulin-like superfamily (ICAM-1, −2, −3, VCAM-1, and PECAM) have been found elevated in SAH-induced vasospasm in both animal and human studies [14]. Increased ICAM-1, expressed in the endothelial layer and the medial layer of the BAs, are correspondent to the severity and timing of vasospasm in experimental SAH in rats [48]. In a rat femoral artery vasospasm study, intraperitoneal administration of ICAM monoclonal antibody significantly decreased the degree of vasospasm and the number of infiltrating leukocytes [27]. Furthermore, administration of a monoclonal antibody against CD11 and CD18, the integrins that interact with ICAM-1, prevented vasospasm in a primate model of vasospasm [36]. Lorenz et al. declared CD45 molecule induces homotypic adhesion of human thymocytes through a ICAM-1-dependent pathway [49]. In this study, treatment with high dose VPA significantly attenuates ICAM-1 and E-selectin in the cortical homogenates of SAH rats, which corresponds to the decreased CD45(+) cells present in the vascular wall of BAs.

Known as regulated on activation, normal T-cell expressed, and secreted (RANTES), CC chemokine ligand-5 is expressed by T-cells, fibroblasts, and mesangial cells and stored in the α-granules of platelets [35]. Once activated, RANTES is deposited onto endothelium and responds to mediate monocytes and T-cells transmigration into the intima [48]. As a T-cell mitogen and mediators of pro-inflammatory cytokines, RANTES has been demonstrated highly expressed in atheroma and atherosclerotic disease [27]. Locati et al’s study also supports through activating a restricted transcriptional program in human monocytes, RANTES exerts a novel recruitment amplification loop of leukocytes and promotes monocyte extravasation and tissue invasion [10]. In this study, high dose VPA is able to restrict RANTES protein expression in SAH induced neuro-inflammation.

The article "Valproic acid attenuates intercellular adhesion molecule-1 and E-selectin through a chemokine ligand 5 dependent mechanism and subarachnoid hemorrhage induced vasospasm in a rat model" was retracted in 2023. Reasons: duplicated images; overlap with earlier publications; unreliable data; concerns about the data.

In summary, the results of this study show that continuous administration of VPA is safe and efficacious in the treatment of vaso-constriction in this experimental model and is meritorious of further investigation. Central nervous system administration of RANTES significantly reversed the anti-vasospasm effect of VPA in the SAH study. Besides, VPA, at an optimal dosage, can attenuate ICAM-1 and SAH related delayed vasospasm through a CCL5 dependent mechanism.

## Conclusions

Despite cerebral vasospasm following SAH has been recognized for more than half a century, the outcome of SAH patients revealed devastating, and stood still after decades of research and treatment on cerebral vasospasm following SAH. Increased evidences revealed there were multifaceted mechanisms contributing to the final pathogenesis. These acuminated results arouse interest to consider the pathogenesis of SAH induced neuro-inflammation and its effect dictates on the patient’s outcome. The breakout of brain blood barrier accompanying SAH may be a critical and complicated pathway underlying the development and maintenance of subsequent vaso-constriction. This study shows that administration of VPA, with its short branch fatty acid, easily penetrates cytoplasm and diminishes SAH induced ICAM-1 and E-selectin as well as CD45(+) cells transmigration into vascular wall in a rodent model of SAH. We suggest that VPA, a HDAC inhibitor, has other effect than anti-convulsion and is useful in treating SAH-induced delayed cerebral ischemia and vasospasm.

## Abbreviations

BA: Basilar artery
caspases: Cysteine requiring aspartate proteases
CCL5: Chemokine ligand 5
CSF: Cerebrospinal fluid
ET: Endothelin
HDAI: Histone deacetylase inhibitor
HRP: Horseradish peroxidase
IEL: Internal elastic lamina
IL-1& -6: Interleukin 1 and 6
ICAM-1: Intercellular adhesion molecule–1
Keap-1: Kelch-like ECH-associated protein 1
NMDA: N-methyl-d-aspartate
Nrf2: Nuclear factor (erythroid-derived 2)-like 2
PBS: Phosphate-buffered saline
SAH: Subarachnoid hemorrhage
TNF-α: Tumor necrotic factor-α
VCAM-1: Vascular cell adhesion molecule–1
VPA: Valproic acid
